This article has been retracted.

# A Nomogram Predicting the Prognosis of Renal Cell Carcinoma Patients with Lung Metastases

**DOI:** 10.1155/2021/6627562

**Published:** 2021-03-18

**Authors:** Xinyu Sheng, Xuan Lu, Jian Wu, Lu Chen, Hongcui Cao

**Affiliations:** ^1^State Key Laboratory for Diagnosis and Treatment of Infectious Diseases, The First Affiliated Hospital, Zhejiang University School of Medicine, 79 Qingchun Rd, Hangzhou City 310003, China; ^2^National Clinical Research Center for Infectious Diseases, 79 Qingchun Rd, Hangzhou City 310003, China; ^3^Zhejiang Provincial Key Laboratory for Diagnosis and Treatment of Aging and Physic-chemical Injury Diseases, 79 Qingchun Rd, Hangzhou City 310003, China

## Abstract

**Background:**

The optimal tool for predicting the survival of renal cell carcinoma (RCC) patients with lung metastases remains controversial.

**Methods:**

We selected patients diagnosed with RCC and lung metastases, from 2010 to 2015, from the Surveillance, Epidemiology, and End Results (SEER) database. After the selection of inclusion criteria and exclusion criterion, the rest of the patients were incorporated into model analysis. Least absolute shrinkage and selection operator (LASSO) regression was used to select the most important features for construction of a nomogram predicting cancer-specific survival. A calibration plot and the concordance index (*C*-index) were used to estimate nomogram efficacy in a validation cohort. The association between important factors selected by LASSO regression, and prognosis was assessed by the Kaplan-Meier (KM) survival curve. The receiver operating characteristic (ROC) curves were drawn to compare sensitivity and specificity between the nomogram we built and the TNM stage-based model.

**Results:**

A total of 1,369 patients met the inclusion criteria, but not the exclusion criteria. The LASSO regression model reduced 15 features to seven potential predictors of survival, including tumor grade, the extent of surgery, N and T status, histological profile, and brain and bone metastasis status. Such features had good discrimination in the KM survival curves. The nomogram showed excellent discriminatory power (*C*-index, 0.71; 95% confidence interval: 0.70 to 0.72) and good calibration in terms of both 1- and 2-year cancer-specific survival. The nomogram showed great discriminatory power (*C*-index 0.68) and adequate calibration when applied to the validation cohort. The areas under the curve (AUCs) of nomogram were 0.767 and 0.780, respectively, and the AUCs of TNM stage were 0.617 and 0.618 at 1 and 2 years, respectively.

**Conclusions:**

Our nomogram might play a major role in predicting the cancer-specific survival of RCC patients with lung metastases.

## 1. Introduction

Renal cell carcinoma (RCC), a common malignant tumor, accounts for 3.7% of all new tumor cases; RCC is more common in male than female patients, and there are 116,000 deaths annually according to the World Health Organization. The most common pathological type (85%) of RCC is clear cell carcinoma [1, 2]. It is important to accurately predict the survival of RCC patients; however, few efficient predictive tools are available [3–5], particularly for patients with metastatic RCC [6] (which remains incurable). Traditionally, immunochemotherapy has been used to treat nonmetastatic RCC, but the response rate was rarely more than 15%. The clinical prognosis of metastatic RCC is poor, and more studies are required [7]. Lung metastasis is the most common metastasis in RCC patients, but few studies have explored the survival of these patients. An accurate predictive tool would improve tumor control and patient quality of life.

The Surveillance, Epidemiology, and End Results (SEER) database (supported by the American National Cancer Institute) contains clinical and pathological data on cancer patients from 19 regions of the United States and is highly representative of the general population. Compared to most previous studies which had small sample sizes, our research relied on the SEER database enhances the credibility of this study.

A nomogram is a readily understood visual tool that transforms a complex regression equation to a simple graph; predictions are thus accessible and of high clinical utility. Nomograms find applications in both medical research and clinical practice [8]. The tumor-node-metastasis (TNM) staging system for RCC has been widely used to predict prognosis, but the clinical utility remains unclear [9–11]. Therefore, we developed a nomogram for predicting the cancer-specific survival (CSS) of RCC patients with lung metastases and compared its ROC curves to that of a TNM staging system-based model. Unlike most previous studies, we used a large patient sample that had been extensively evaluated and documented.

## 2. Materials and Methods

### 2.1. Patients

Data were obtained from the SEER database. The SEER database covers almost 28% of the US population and is the largest cancer database in the US. All cases are derived from the SEER Program (http://www.seer.cancer.gov) SEER^∗^Stat database (version 8.3.5, accession number: 12099-Nov2018). Abundant information is available, including patient demographics and cancer characteristics. A total of 89,382 patients (including 12,187 stage M1 patients) were newly diagnosed with RCC from 2010 to 2015. The inclusion criteria were as follows: (1) RCC patients from 2010 to 2015 in the US and (2) combined with lung metastases. Thus, we included 1,369 RCC patients with lung metastases in the analysis (Figure 1). Exclusion criteria were as follows: history of other tumors (begin or malignant), age<18, and rare pathological features and data with incomplete information. The following five pathological types of RCC accounted for more than 90% of all cancers: clear cell, papillary, chromophobe, and sarcomatoid RCCs and collecting duct carcinoma (CDC). We excluded patients with other types of carcinoma.

### 2.2. Clinicopathological Features

The following data were collected: years at diagnosis and evaluation, age, race, sex, extent of surgery (none, partial nephrectomy (PN), or radical nephrectomy (RN)), tumor histology, histological grade, nodal (N) stage, insurance and marital status, laterality, tumor size, CSS, and follow-up duration. There were four histological grades (I–IV). Marital status was classified as “unmarried” (including “single (never married)” and “unmarried”), “married” (including “married under common law”), and “no longer married” (“widowed”, “separated”, and “divorced”). The median survival time was 10 months, and the maximum survival time was 70 months.

### 2.3. Survival Analysis and Statistical Methods

The primary outcome was the survival time (from hospital admission to the date of death or last follow-up). Clinicopathological features are summarized as median values with interquartile range (IQR), or as frequencies with percentages, for both the training and validation cohorts. The associations of the factors selected from the least absolute shrinkage and selection operator (LASSO) regression analysis with CSS were evaluated by drawing Kaplan-Meier curves. A nomogram was created based on the results of the LASSO regression. Discriminatory power was quantified using the concordance index (*C*-index). The “rms” R package was used to evaluate the nomogram and draw calibration curves. All statistical analyses were performed using R software (ver. 3.5.3; R Foundation for Statistical Computing, Vienna, Austria). All tests were two-sided and a *P* value < 0.05 was considered statistical significance.

## 3. Results

### 3.1. Clinicopathological Characteristics

Of the 6,685 RCC patients who developed lung metastases from 2010 to 2015, 1,369 were included in the final analysis (976 in the training cohort and 393 in the validation cohort; Table 1). We considered the three major types of metastases (the brain, bone, and liver). The gross pathological types were clear cell, papillary, chromophobe, and sarcomatoid RCCs and CDC. The median age of both cohorts was 60 years, where RCC is more common in the elder. The median follow-up time was 10 months (range: 1–70 months) and the 1- and 2-year CSS rates were 53.9 and 34.8%, respectively.

### 3.2. Feature Selection and Prognostic Signature Building

We reduced the initial 15 features of the 976 patients in the training cohort to seven potential predictors of survival: T status (coefficient, 0.106) N status (coefficient, 0.440), tumor grade (coefficient, 0.211), extent of surgery (coefficient, -0.490), pathology (coefficient, 0.120), and brain and bone metastasis status (coefficient, 0.581 and 0.464) (Figure 2). Feature selection was performed using a LASSO binary logistic regression model. Dotted vertical lines were drawn at the optimal values (derived using the minimal criteria with one standard error (the “1-SE” criteria), see Figure 1). The final *λ* value was 0.068 and the log (*λ*) value was -2.687. We included the coefficient profiles of all 15 features in the diagram.

### 3.3. Kaplan-Meier Curves of Significant Features

All seven potential predictors of survival were found to be useful for predicting CSS in the training cohort (Figure 3). It was clear that patients lacking metastases had better CSS, which was also significantly enhanced by PN or RN. Patients receiving operation (either PN or RN) had a better CSS than those who did not. Not surprisingly, lymph node metastasis could not afford a significant survival benefit. The significant differences in tumor grade and histology among RCC types also affected the CSS outcomes.

### 3.4. A Prognostic Nomogram for CSS

The prognostic nomogram comprising all factors that significantly affected CSS is shown in Figure 4. The *C*-index for CSS prediction was 0.71 (95% confidence interval: 0.70 to 0.72). The calibration plots for the 1- and 2-year survival probabilities of RCC patients with lung metastases revealed excellent agreement between prediction and observation in training cohort (Figures 5(a) and 5(b)).

### 3.5. Validation of Predictive Accuracy

The follow-up time in the validation cohort was 10 months (range: 1–67 months) and the 1- and 2-year CSS rates were 56.3 and 43.1%, respectively. The *C*-index of the nomogram for CSS prediction was 0.68. The calibration plots of the survival probability of the validation cohort, for 1 and 2 years after RCC diagnosis, revealed good agreement between prediction and observation.

### 3.6. ROC Comparison with TNM Stage

We then applied the time-dependent ROC curves to compare sensitivity and specificity between the nomogram we built and the TNM stage at 1 and 2 years. The areas under the curve (AUCs) of nomogram were 0.767 and 0.780, respectively, and the AUCs of TNM stage were 0.617 and 0.618 at 1 and 2 years, respectively (Figure 6).

## 4. Discussion

In a LASSO regression, seven prognostic factors for RCC patients with lung metastases were identified, based on which a nomogram was constructed including tumor grade, extent of surgery, T and N status, histology, and brain and bone metastasis status. This was used to predict 1- and 2-year CSS in a large cohort of metastatic RCC patients drawn from the SEER database. The nomogram was validated, internally and externally, in terms of its discriminatory power and calibration.

There exist several outcome prediction models for RCC patients, though none of them is developed for patients with lung metastases. Due to the natural differences in tumor microenvironment, models set for metastatic and nonmetastatic RCC are different. The stage, size, grade, and necrosis (SSIGN) score and the University of California Los Angeles Integrated Staging System (UISS) are two widely used tools for prognosis prediction [12, 13]. SSIGN score is calculated to divide localized RCC patients into three groups and to predict 5-year metastasis-free survival rate. UISS can be used to predict 5-year disease-specific survival for both metastatic and nonmetastatic RCC patients, which includes T stage, Fuhrman's grade, and ECOG (Eastern Cooperative Oncology Group) status. Besides the two common tools for prediction, other three prognostic models are performed in the previous studies [14–16].

As for metastatic RCC, prediction tools are used for either selecting those patients who might benefit from adjuvant treatment or predicting survival rate. The patients care more about their survival time. Previous studies have launched some prediction models based on demographic and tumor pathology information [17, 18]. However, most of them just proposed prognostic factors, rather than integrating them into scores and presenting them in a concise form.

The effect of lung metastases on prognosis in RCC patients remained controversial. A research with 782 patients from Groupe Français d'Immunothérapie took diverse metastatic sites including the lung, mediastinum, bone, and liver into consideration, and the results showed that only the lung metastasis was not associated with overall survival [19]. Similarly, a retrospective study showed that the overall survival did not differ between patients with less than 8.5 months and more than 8.5 months [20]. However, as lung metastasis is the most common metastasis in RCC patients, it is hard to say that it has no effect on the overall survival of RCC. This can be corroborated by a study on adult metastatic RCC that lung metastasis together with weight loss and disease-free interval resulted in a worse survival [21]. Also, although there were several prognostic tools for RCC patients with lung metastasis, none of them was developed for RCC patients with lung metastases, which is exactly what we want to do in this study.

Currently, only few dedicated models predict the overall survival (OS) or CSS of RCC patients, particularly those with metastases. A model based on the TNM staging system is currently the default clinical model, and it evaluates tumor size and local extension of the primary tumor (T), regional lymph node involvement (N), and distant metastasis status (M) [22, 23]. Because we evaluated metastatic RCC patients, T and N status were retained in our nomogram. Although the TNM-based model is widely used to predict the survival of RCC patients, it is unclear whether the model is appropriate. A few studies found that models based on the TNM staging system were inaccurate in terms of predicting the RCC survival rate [24]. One study even reported no association between TNM staging system data and RCC patient outcomes. A study of more than 500 nonmetastatic RCC patients found that the prognostic utility of the TNM staging system was limited [25]. Few studies have focused on metastatic RCC; it is essential to establish a novel tool for predicting the outcomes (especially survival rates) of metastatic RCC patients. Most RCC metastases are in the lungs; these patients require special attention. The TNM staging system is clearly biased, emphasizing pathological indicators over other, such as clinical and treatment characteristics, which are more important from our perspectives.

We searched all the metastatic RCC prognostic models and compiled them into Table S1 in the Supplementary Material. Among these models, “performance status,” “signs of inflammation,” and some biochemical indicators including ALP, calcium, LDH, hemoglobin, and WBC count were not included in the SEER database, which is one limitation of analysis. However, although these models were developed for a while, none of them was compared with the traditional TNM staging system, which is worth to be taken into consideration. The nomogram we developed exhibited great discriminatory power and the CSS of the training and validation cohorts were well-calibrated. It proved that this prognostic model is stable and convincing. Also, we concerned the two types of surgical methods, PN and RN, since they might affect the patients' perioperative state and therefore affect the survival of RCC patients with lung metastases.

A nomogram is an intuitive visual tool for predicting disease survival and can be used to explain survival probability to patients in a straightforward manner. Many authors now use nomograms to predict disease (including RCC) survival rates [26, 27]. Nomograms containing more information than the TNM staging system; they better predict the outcomes of patients with pancreatic and hepatic carcinoma [28, 29] and RCC. We considered seven factors including pathological type and clinical and treatment characteristics, to minimize bias when predicting prognosis.

The strengths of our study were as follows. First, our nomogram is the only tools effective for predicting the CSS of RCC patients with lung metastases among existing models. Indeed, it is an effective bridge connecting doctors and patients. Second, we focused on a specialized cohort, i.e., RCC patients with lung metastases (the most common metastasis in these patients). Third, our study is a good representative of the general population. The SEER database we used covers the entire United States and is thus much larger and more comprehensive than single-center databases; this feature enhances the credibility of our study.

This study also had some limitations. First, our research lacks external validation, though the SEER database compensates for the homogeneity of patients from single research center to some extent as it covers millions of patients all around US. Second, as the study was retrospective in nature, patient allocation to the training and validation cohorts may have been biased; randomized control trials are needed. Third, some biochemical indicators including ALP, calcium, LDH, hemoglobin, and WBC count were not included in the SEER database and the discriminatory power of our nomogram could not be compared with other prognostic models. Also, a larger cohort would have allowed us to detect small differences between patient subgroups. Finally, unknown factors may affect the CSS of RCC patients with lung metastases. More data are needed to confirm the effectiveness of the nomogram; to this end, a prospective study is planned.

## 5. Conclusion

The novel prognostic model based on the SEER database could predict the cancer-specific survival of RCC patients with lung metastases.

## Figures and Tables

**Figure 1:** Flow chart of patient selection.

**Figure 2:** Feature selection using a least absolute shrinkage and selection operator (LASSO) regression model. (a) Tuning parameter (*λ*) selection for the LASSO model involved fivefold cross-validation using the minimal criteria. Dotted vertical lines were drawn at the optimal values; one standard error was added to each criterion to yield the 1-SE criteria. (b) The LASSO coefficients of the 15 features.

**Figure 3:** Kaplan-Meier curves of selected features. Seven features were included in the final model. The cancer-specific survival of renal cell carcinoma (RCC) patients with lung metastases was predicted by T status (a), N status (b), tumor grade (c), extent of surgery (d), pathology (e), brain metastasis status (f), and bone metastasis status (g).

**Figure 4:** The prognostic nomogram. The nomogram was developed using the training cohort. The seven features selected by LASSO regression included T status, N status, tumor grade, extent of surgery, pathology, brain metastasis status, and bone metastasis status. The nomogram accurately predicted 1- and 2-year survival.

**Figure 5:** Calibration curves of the prognostic nomogram for each cohort. (a) Calibration curve of the nomogram for the training cohort at 1 year. (b) Calibration curve of the nomogram for the training cohort at 2 years. (c) Calibration curve of the nomogram for the validation cohort at 1 year. (d) Calibration curve of the nomogram for the validation cohort at 2 years.

**Figure 6:** Time-dependent receiver operating characteristic (ROC) curves of the nomogram score and model based on TNM stage for CSS of RCC patients with lung metastases. (a) ROC at 1 year. The areas under the curve (AUCs) of the nomogram and TNM stage were 0.767 and 0.617, respectively. (b) ROC at 2 year. The areas under the curve (AUCs) of the nomogram and TNM stage were 0.780 and 0.618, respectively.

**Table 1:** Clinicopathological characteristics of RCC patients with lung metastases.

Characteristic	Primary cohort (*n* = 976)		Validation cohort (*n* = 393)		*P* value
	No. of patients	%	No. of patients	%	
Age (years)					0.72
Median	60		60		
Range	54-68		54-68		
Sex					0.252
Male	705	72.2	271	69	
Female	271	27.8	122	31	
Race					0.937
White	831	85.1	335	85.2	
Black	64	6.6	24	6.1	
Other	81	8.3	34	8.7	
Grade					0.928
I	29	3	10	2.5	
II	188	19.3	77	19.6	
III	405	41.5	158	40.2	
IV	354	36.3	148	37.7	
Laterality					1
Left	480	49.2	193	49.1	
Right	496	50.8	200	50.9	
T					0.859
T1a	19	1.9	6	1.5	
T1b	82	8.4	29	7.4	
T2a	89	9.1	43	10.9	
T2b	83	8.5	36	9.2	
T3	572	58.6	224	57	
T4	131	13.4	55	14	
N					0.875
N1	304	31.1	120	30.5	
N0	672	68.9	273	69.5	
Surgery					0.659
No surgery	231	23.7	84	21.4	
PN	19	1.9	8	2	
RN	726	74.4	301	76.6	
Tumor size (mm)					0.356
Median	95		100		
Range	75-120		75-120		
Pathological type					0.582
pRCC	28	2.9	12	3.1	
ccRCC	697	71.4	288	73.3	
RCC, NOS	168	17.2	53	13.5	
sRCC	8	0.8	3	0.8	
chRCC	63	6.5	30	7.6	
CDC	12	1.2	7	1.8	
Brain metastasis					0.421
Yes	116	11.9	40	10.2	
No	860	88.1	353	89.8	
Bone metastasis					<0.001
Yes	116	11.9	78	19.8	
No	860	88.1	315	80.2	
Liver metastasis					0.523
Yes	131	13.4	47	12	
No	845	86.6	346	88	
Insurance status					0.93
Yes	936	95.9	378	96.2	
No	40	4.1	15	3.8	
Marital status					0.115
Unmarried	155	15.9	57	14.5	
Married	642	65.8	280	71.2	
Negative married	179	18.3	56	14.2	

Abbreviations: ccRCC: clear cell renal cell carcinoma; pRCC: papillary renal cell carcinoma; chRCC: chromophobe renal cell carcinoma; sRCC: sarcomatoid renal cell carcinoma; CDC: collecting duct carcinoma.

## Data Availability

The data used to support the findings of this study are included within the article.

## Supplementary Materials

Supplementary Materials Supplementary Table S1: characteristics in various prognostic models for metastatic RCC.
